# Predicting Mental Health Problems with Automatic Identification of Metaphors

**DOI:** 10.1155/2021/5582714

**Published:** 2021-04-30

**Authors:** Nan Shi, Dongyu Zhang, Lulu Li, Shengjun Xu

**Affiliations:** ^1^School of Software, Dalian University of Technology, Dalian 116620, China; ^2^Psychological Health Education and Counseling Center, Dalian University of Technology, Dalian 116620, China

## Abstract

Mental health problems are prevalent and an important issue in medicine. However, clinical diagnosis of mental health problems is costly, time-consuming, and often significantly delayed, which highlights the need for novel methods to identify them. Previous psycholinguistic and psychiatry research has suggested that the use of metaphors in texts is linked to the mental health status of the authors. In this paper, we propose a method for automatically detecting metaphors in texts to predict various mental health problems, specifically anxiety, depression, inferiority, sensitivity, social phobias, and obsession. We perform experiments on a composition dataset collected from second-language students and on the eRisk2017 dataset collected from Social Media. The experimental results show that our approach can help predict mental health problems in authors of written texts, and our algorithm performs better than other state-of-the-art methods. In addition, we report that the use of metaphors even in nonnative languages can be indicative of various mental health problems.

## 1. Introduction

Mental health problems have become increasingly serious. They not only endanger people's physical and mental health, but also affect the development of the country and society. The WHO survey (https://www.who.int/health-topics/mental-health) shows that about 13% of people worldwide suffer from mental disorder, which cost the global economy one trillion dollars each year. Depression is one of the main causes of disability. Suicide is the second leading cause of death among children aged 15–29. About 20% of children and adolescents in the world suffer from mental illness, and the highly educated population also suffer from psychological distress which affects their academic performance [1–3]. However, clinical diagnosis of mental health problems is costly, time-consuming, and often significantly delayed, which highlights the need for novel methods to identify these conditions.

Metaphorical expressions are frequently used in human language [4–7]. They involve both linguistic expression and cognitive processes [8] and are an implicit way to convey emotions [9–11]. Human emotions and mental state, which are important for mental health, are frequently communicated and expressed through metaphors. This suggests that the use of metaphorical expressions in texts may indicate mental and cognitive status and so help in mental health screening.

Psycholinguistic and psychiatry studies have indicated that the use of metaphors in texts is linked to the mental health illness of their authors [12–16]. For example, patients with schizophrenia may metaphorically use the phrase “time vessels” to refer to watches and “hand shoes” to refer to gloves. In other words, the use of metaphor in individuals with mental illness may differ from those without, which could offer new opportunities to identify mental illness using metaphors as a diagnostic indicator. Although it is not clear what causes these deviations in metaphor production, neuroscience research offers some clues. Scholars note that some mental illnesses such as schizophrenia relate to dysfunction of the amygdala, which processes and regulates emotion [17]. Other research suggests that metaphorical texts are associated more with activation of the amygdala than with areas relating to literal speech [18].

With the development of artificial intelligence and various data processing technologies [19–25], the efficiency of modern medical diagnosis is constantly improving. As an important part of artificial intelligence, natural language processing is widely applied in mental health related issues [26–28]. Shatte et al. [29] reviewed the application of machine learning in mental health: four main application areas, including detection and diagnosis [30, 31]; prognosis, treatment, and support; public health; research and clinical management. The most common mental health conditions addressed include depression, schizophrenia, and Alzheimer's disease. Prior work has shown the feasibility of using NLP techniques with various features extracted from text messages such as linguistic, demographic, and behavioral features to predict mental illness such as depression [32], suicidality [33], and posttraumatic stress disorder [34]. However, few studies have involved the application of metaphor, a deep semantic feature, as a means of detecting and predicting mental health problems. Along with the rapid explosion of social media applications such as Twitter and Facebook, there seems to be a significant increase in metaphorical texts on a variety of topics, including products, services, public events, and tidbits of people's lives. It seems to be an important and promising challenge to leverage metaphor features for supporting the identification and prediction of mental health problems.

In this paper, we propose the use of automatically detected metaphors in texts to predict various mental health problems including anxiety, depression, inferiority, sensitivity, social phobias, and obsession. We named our method Metaphor-Sentiment Model (MSM) and we performed experiments on a compositional dataset we created from second-language student essays and the eRisk2017 dataset collected from Social Media. Our contributions are as follows.

- We propose a novel approach to identify several mental health problems by using linguistic metaphors in texts as features. To the best of our knowledge, we are the first to leverage metaphor features for supporting the identification and prediction of mental health problems.
- The experimental results show that our proposed approach can help predict the mental health of authors of written texts and our algorithm gives fairly good performance, compared to state-of-the-art methods.
- The work shows how semantic content, specifically usage of metaphors in writings produced by individuals, can help in detection of six mental health problems. This seems to be a new result where usage of metaphors even in nonnative languages can be used as indicative of various mental health problems.
- We contribute to a novel, scarce, and valuable dataset, which will be released publicly, consisting of second-language speakers' essays and data on authors' mental health problems obtained from a psychological survey.
- Due to the scarcity of relevant work, exploring features that influence mental health using computational approaches can potentially help with early detection and treatment of mental health and related problems.

## 2. Related Work

### 2.1. Mental Health in NLP

NLP techniques have been applied to speculate on people's mental health status, based on written texts, such as those on Facebook, Twitter, etc., and they can be used to obtain information on the user's psychological state directly and efficiently [35]. In recent years, scholars have explored many different features of various datasets to explore the mental health status that lies behind a text. Nguyen et al. [36] used data from the foreign Live Journal Post website to collect 38 k posts from the mental illness community and 230 k posts from mentally healthy communities for mental illness prediction. They tried various approaches, including linguistic inquiry and word count (LIWC), which obtain features of language, social, effective, cognitive, perceptual, biological, relativistic, personal attention, and oral, emotional feature (also based on LIWC) and latest dirichlet allocation (LDA) topic models, ultimately achieving 93% accuracy. Franco-Penya and Sanchez [37] built a tree structure based on the n-grams feature and combined other features and support vector machine (SVM) learning methods to design classifiers to detect mental health status in CLPsych2016 [38]. Cohan et al. [39] comprehensively considered lexical features, contextual features, textual data features, and textual topical features on the same dataset, using SVM classifiers to complete detection tasks. Ramiandrisoa et al. [40] tried a variety of lexical features in another evaluation task on the CLEF 2018 eRisk database [41], including bag of word models, specific category words, and special word combinations, and they converted text into vectors for classification. Weerasinghe et al. [42] investigated language patterns that differentiate individuals with mental illnesses from a control group, including bag-of-words, word clusters, part of speech n-gram features, and topic models to understand the machine learning model.

In addition to the use of text and other user characteristics, the rise of deep learning has provided new ways to detect mental illness through text. Benton et al. [43] modeled multiple scenarios to predict different suicide risk levels and built a multitasking learning framework (MTL) to meet the needs of different tasks. Trotzek et al. [44] first converted text into vectors and then completed classification task through a convolutional neural network to predict the mental health status of the user. Sekulic and Strube [45] applied a hierarchical attention network and analyzed phrases relevant with social media users' mental status by inspecting the model's word-level attention weights. Multimodal thinking is also applied in mental health research [46, 47]. They used a multimodal approach that consists of jointly analyzing text and visual and audio data and their relation to mental health more than text analysis.

### 2.2. Datasets

As discussed above, metaphorical expressions are associated with mental and cognitive status. Since a metaphor involves cognitive processes, it may be feasible to screen and monitor mental and affective status no matter the degree of fluency in the language. We thus assume that metaphor is an important textual feature for mental health detection among language users, including both native and second-language speakers. We collected data from two different sources to verify our assumptions and increase the reliability of our experiments in this study of the relationship between metaphor use and mental health status.

### 2.3. Student Composition and Mental Health

We collected English composition data from English-proficient Chinese college students who speak English as a second language. We also collected mental health data from these students using a psychological survey. First, we used online and offline campus advertisements to recruit 164 college freshman participants who passed the national college students' English level 4 test in China, which means they are native Chinese and fluent in English writing. Prior to participation, all participants provided a consent form indicating their willingness to take part in the study. Participants provided their personal information via a questionnaire and then wrote a composition with 500 English words or more within a two-hour period. The composition had two parts: described their previous life experience and then presented their future plans, including their ideal future lives, thoughts on life, targets for their future lives, and plans to overcome barriers. The content gave us a deep understanding of their psychological states [48], which is essential for the detection of mental health problems.

After writing their composition, students were required to complete a mental health questionnaire that assessed two levels of mental health problems. The first level involved is serious mental health problems, mainly serious psychoses such as hallucinations, suicidal behavior, and suicidal inclination. In our survey, only a few students had first-level problems. The second level involved common mental problems, such as anxiety, depression, inferiority, sensitivity, and social phobias. Mental problems were assessed on the basis of the standard score for screening indexes. Specifically, participants were assessed with mental health problems when their scores on certain indexes exceeded typical results. We excluded data from 8 students because we could not match their mental problems with fuzzy indexes from their mental health data. Effective mental health data for the remaining 156 students is presented in Table 1. Meanwhile, we extracted data from students without mental health problems to use as controls for analyzing differences in metaphor use with sentiment features in texts.

The process of data collection lasted four months and resulted in a total of 156 compositions with 130,044 words from 156 students (aged 18–23 yrs, mean = 19.06 yrs, SD = 0.19, males = 86, and females = 70), together with mental health data obtained from the psychological questionnaire. These data were kept secure and stored with no identifying factors, i.e., consent forms and questionnaires.

### 2.4. eRisk2017 Data

The eRisk2017 task on early risk detection of depression [49] provides a dataset containing posting contents and comments from Reddit. The task identified 135 Reddit users with depression and 752 Reddit users without depression through their posts and comments. The word quantity for each Reddit user varies from 10 to 2,000. The dataset for each Reddit user contains individual identification, writing data, text title, writing type, and writing contents. Paper [50] details the construction of the eRisk data. They first selected Reddit from multiple social media and collected the post of depression diagnosis through specific search (such as I was diagnosed with depression). Posts are manually evaluated to identify users who are really diagnosed with depression. They collected patients' text records published on Reddit over a period of time. We combined the contents for each Reddit user in chronological order for the present study.

## 3. Methodology

Our work flow is shown in Figure 1. Metaphor is linked to the mental health problems as described above. We extracted metaphors from texts and designed metaphor feature sets to predict various mental health problems. Our method also considered sentiment features in the sample texts as this feature has been widely used in mental health research [14, 44, 51, 52]. We applied metaphor and sentiment features in our Metaphor-Sentiment Model (MSM) to predict mental health problem. The feature extraction algorithm is briefly summarized in algorithm 1, and more details will be introduced below.

### 3.1. Metaphor Feature Extraction

For metaphor-based features, we considered the following (Algorithm 1, Step 1):

- The percentage of tokens tagged as metaphor by the automatic metaphor identification method
- The probability of a sentence containing metaphor

We also considered the sentiment of metaphor expressed in a sentence that is consistent with the sentence sentiment. First, SentiStrength (http://sentistrength.wlv.ac.uk/) was used to analyze the overall sentiment of a sentence. SentiStrength analysis yields two scores for sentiment strength: negative (scores −1 to −5) and positive (scores 1 to 5). The sum of the two values is the overall sentiment score for the sentence. A sentiment score of 0 is defined as neutral. Next, we determined sentiment of metaphor using three specific feature values (Algorithm 1, Step 3):

- The number of metaphors with positive sentiment (positive sentiment score)
- The number of metaphors with negative sentiment (negative sentiment score)
- The average sentiment score for all metaphors

In our method, metaphors were identified automatically using a technique that has shown the best performance for token-level metaphor identification tasks to date [53]. The automatic metaphor identification system contains four steps: (1) it trains word embeddings on a Wikipedia dump based on Continuous Bag of Words (CBOW) and Skip-Gram models to obtain input and output vectors for every word; (2) it selects detected words to assess metaphoricity and separates the detected words from a given sentence; (3) it extracts all possible synonyms and direct hypernyms, including their inflections, of the detected word from WordNet, and it adds them to the candidate word set *w*, which contains all possible senses of the detected word; and (4) it selects the best fit word *w*^*∗*^, which represents the actual sense of the detected word in the a given sentence, from the candidate word set *w*, using the following formula:

(1) $$\begin{array}{c} w^{*}=\text{arg}\underset{k}{\max}\text{SIM}\left(v_{k},v_{\text{context}}\right), \end{array}$$

where *k* ∈ *w*, *v*_*k*_ is the input vector of the CBOW or Skip-Gram entry for a candidate word *k*, and *v*_context_ means the average of all input vectors for context words. The best fit word has the highest cosine similarity with the context words. Finally it computes the similarity value for the detected word and the best fit word using output vectors to measure the difference of sense between the detected word and the context. The detected word is labeled as metaphorical when the similarity value is less than the given threshold. In practical applications we detected every content word in the sentence. The detailed process is presented in Algorithm 2.

We trained and tested the identification algorithm on a metaphor dataset developed by Mohammad [10] that contains 210 metaphorical sentences whose detected words are annotated manually with at least 70% agreement. We selected the same number of literal sentences from thousands of literal sentences in the dataset. The best metaphor identification performance had a precision of 0.635, recall of 0.821, and F1 value of 0.716 with a threshold of 0.5, which matches the identification performance reported by Mao [53].

For evaluating the performance of the metaphor identification method with our dataset, we randomly selected ten compositions from each of the seven groups that correspond to six mental health problems and healthy control. In total, seventy compositions were analyzed. The metaphor identification performance using the student dataset had a precision of 0.632, recall of 0.935, and F1 value of 0.754.

Figure 2 shows examples of metaphors detected by the automatic metaphor identification method from the student composition dataset (a-c) and eRisk2017 dataset (d-f). The sentences match two words from different domains: for example, a source word tagged as metaphorical, such as *broken*, and a target word such as *dream*. However, this token-level metaphor identification algorithm produces some errors since it identifies a metaphor based on local information around the detected word and cannot effectively recognize fixed collocation. For example, in the phrase *I ultimately got up on my own*, the algorithm mistakenly tags the word *own* in *on my own* as metaphorical.

### 3.2. Sentiment Feature Extraction

The sentiment feature set included the average value of the five dimensions of all words; the proportion of positive sentences, negative sentences, and neutral sentences; the average emotional score of the sentences, and the emotional fluctuation value of each article, yielding ten specific features in total.

We used SentiStrength to obtain sentiment scores for sentences in the texts as above, in order to calculate the proportion of positive sentence, negative sentence, and neutral sentence; the average sentiment score of the sentences of article; the sentiment fluctuation score of each article (Algorithm 1, Step 2).

The average score of the sentences in each article was calculated to determine the emotional value of the article using the following formula:

(2) $$\begin{array}{c} E=\frac{\sum_{i=1}^{n}S_{i}}{n}, \end{array}$$

where *E* represents the average sentiment value of the text, *S*_*i*_ represents the emotional score of the *i* th sentence, and *n* is the number of the sentences in the text. And the fluctuation score is obtained by subtracting the emotional scores of two consecutive sentences in the article and taking the absolute value. We used the average as its sentiment fluctuation value. It is determined by the following formula:

(3) $$\begin{array}{c} F=\frac{\sum_{i=2}^{n}\left|S_{i}-S_{i-1}\right|}{\left(n-1\right)}, \end{array}$$

where *F* represents the emotional fluctuation value of the text.

Scores for the five dimensions (values of pleasantness, attention, sensitivity, aptitude, and polarity) were obtained using SenticNet (http://www.sentic.net) (Algorithm 1, Step 4). The averages of the five dimensions of all words were taken as an indicator of the article's emotions. Averages were calculated as this example for pleasantness values:

(4) $$\begin{array}{c} P=\frac{\sum_{i=1}^{n}W_{i}}{n}, \end{array}$$

where *P* represents the average for pleasantness values and *W*_*i*_ represents the pleasantness value of the *i* th word. Averages for attention values, sensitivity values, aptitude values, and polarity values were computed similarly.

## 4. Metaphor Analysis

We analyzed metaphor use for six mental problems and health control based on automatic identified result, including examples of identified metaphors and statistical analysis.

Table 2 shows examples of the most frequently used metaphors for each of seven mental health groups. In order to demonstrate characteristics of each group, we excluded the metaphorical words, which occurred with the most frequency in all mental health groups, such as *pay*, *top*, and *limit*. The same metaphor word was often used in a different way by those in the mentally healthy group compared to those in mental health problem groups, as illustrated in the following examples:

 
*Ex1. Teachers always try their best to meet the requirements of students*.
 
*Ex2. We always meet various difficulties on the way to study.*

The sentence in the first example was taken from a composition by a student in the healthy control group and expresses a positive sentiment, while the second example was taken from a composition by a student in depression group and expresses a negative sentiment.

We study the emotion of text and effect of metaphor in Student Composition data. The statistical information is shown in Table 3.

Avg. emotion denotes average score of emotion of all text and meta emotion is average emotional score of sentence with metaphor. People in sensitivity group have highest emotional score and that of obsession group is lowest. Meta emotion overall is 0.05 lower than avg. emotion, which shows that, in Student Composition Dataset, students are more likely to express negative emotions and describe sad things through metaphor, for example, sentences A and C in Figure 2.

  Ex3. My dream was broken
  Ex4. He will walk into society eventually

The former expresses the lost mood of broken dream, and the latter is used to show the helpless mood of growing up and entering the society. Both of them apply metaphor to express negative emotions.

To better understand the characteristics of metaphor use for each mental problem, we labeled students as *sick* or *not sick* for every particular mental problem and analyzed metaphor features between the two groups. The histograms in Figure 3 show the situation of different metaphor features for each mental health problem. We found that the probability of a sentence containing metaphor was higher among students with inferiority or social phobia than students without these mental problems (*t* = 1.775, *p* < 0.1; *t* = 1.695, *p* < 0.1). Students with social phobia were more inclined to use metaphors with negative sentiments than students without social phobia (*t* = 1.978, *p* < 0.05). Additionally, students with obsession had significantly lower scores for average sentiment value of metaphor than students without obsession (*t* = −2.060, *p* < 0.05). The most distinguishing index of compositions by students with mental health problems was the probability of sentence with metaphor. Students with mental health problems had higher eigenvalues for this variable than those in the healthy group.

## 5. Experiments

We compared the predictive performance of MSM and baseline on the eRisk2017 dataset [49] and on the second-language speaker essays dataset, and we evaluated the metaphor feature with common text features used in baseline. Each of the six mental health problems in the second-language speaker dataset was subjected to a separate bicategorization task. We planned to verify the effectiveness of metaphorical features in the detection of various mental health problems, and we used the same Metaphor-Sentiment feature set in each mental health problem prediction task. Different model parameters will be obtained for different mental problems to deal with metaphorical features.

We applied Synthetic Minority Oversampling Technique (SMOTE) to alleviate the imbalance between positive and negative samples on Student Composition dataset. SMOTE algorithm analyzes samples of minority and produces new samples to the dataset. The specific process: (1) randomly select a sample *x* from minority and calculate the Euclidean distance between it and other samples in this category; (2) randomly select a sample *x*_*n*_ from the *k* nearest neighbors of *x* calculated in the previous step; (3) according to the following formula, a new sample is constructed and added to the minority sample set; (4) repeat the above steps until the appropriate sample size is obtained.

(5) $$\begin{array}{c} x_{\text{new}}=x+\text{rand}\left(0,\;1\right)*\left|x-x_{n}\right|. \end{array}$$

### 5.1. Baseline

The prediction method proposed by [44] was chosen as a baseline since it showed the best performance in eRisk2017 and eRisk2018. They applied two methods to the eRisk2017 dataset to detect people suffering from depression. One method involved logistic regression using features extracted by four word frequency statistics tools—LIWC (http://liwc.wpengine.com/), NRC Emotion Lexicon (http://www.saifmohammad.com/WebPages/NRC-Emotion-Lexicon.htm), Opinion Lexicon (http://www.cs.uic.edu/∼liub/FBS/opinion-lexicon-English.rar), and VADER Sentiment Lexicon (http://www.nltk.org/_modules/nltk/sentiment/vader.html). These tools scan the input text to calculate the frequency of words in different categories, such as the normalized frequency of positive words—words used for expressing positive emotion. The output statistics of word frequency can be transferred into the classifier as text features. The other was a deep learning-based method that employed a convolutional neural network (CNN). We reproduced both methods and compared them with our method for the two datasets.

### 5.2. Prediction Method

We used a metaphor-based feature set and a sentiment-based feature set to build Metaphor-Sentiment Model (MSM) for predicting mental health status. We compared the performance of three common classifiers: logistic regression, SVM, and neural network. The neural network produced the best results as the relationship between features and mental health problems may be nonlinear. In order to prevent the neural network model from overfitting in training small-scale student dataset, we added L2 regularization, dropout layer, and early-stop mechanism to the model. Meanwhile, the number of layers and hidden layer nodes in the network are determined by testing. 10-fold cross validation is applied in experiment to ensure the performance of model.

The neural network in this paper was built using Keras (https://github.com/keras-team/keras), which is a four-layer, fully connected neural network comprising one input layer, two hidden layers, and one output layer. The input layer was the vector that combined the metaphorical features and sentiment features extracted from the data. The two hidden layers had output dimensions of 100 and 50, respectively. The input layer and the two hidden layers used concatenated rectified linear units (CReLU) for the activation function. We added a dropout layer between two hidden layers with a dropout rate of 0.4 to avoid overfitting. The output layer used Softmax for the activation function, which yielded a generalization of logic functions and output vectors with two dimensions.

### 5.3. Experiment Performance

The eRisk2017 dataset has been divided into a training set and a test set [49]. We tested MSM using either a sentiment-based feature set, a metaphor-based feature set, or both and compared the results with those using the baseline method. The results are shown in Table 4. Our identification method outperformed the two baseline methods in terms of both accuracy and F1-score. In addition, the results indicate that metaphor-based feature sets are helpful for detecting depression. These results demonstrate the superiority of our prediction method compared with established methods such as those used for our baseline.

We used 10-fold cross validation to partition our composition dataset collected from second-language students to evaluate the prediction performance of MSM compared to the baseline methods. The results are shown in Tables 5 and 6.

Table 5 compares the accuracy of the two baseline methods with that of our method for the prediction of six mental health problems. The results show that MSM obtained the highest accuracy, with an average accuracy for all six mental health problems that was significantly higher than baseline (Fisher's exact test: *p* < 0.05), especially with regard to the sensitivity prediction task (Fisher's exact test: *p* < 0.005). The metaphor-based feature set played an important role in MSM and outperformed the sentiment-based feature set for all mental health group prediction tasks. It achieved the highest accuracy for predicting inferiority, which corresponds to the significant difference in metaphor use between students with inferiority and those without inferiority, as discussed above.

Considering the unbalanced samples, we also computed the F1-score for all mental health problem prediction tasks. The results are shown in Table 6. Overall, using all feature sets, our method showed the highest performance for prediction of the six mental health problems in terms of the average F1-score. The improvement in F1-score was significant with respect to students with sensitivity (Fisher's exact test: *p* < 0.05). The logistic regression baseline method achieved the same results as our method overall. The metaphor-based feature set from our method showed the highest F1-scores for predicting inferiority and social phobia.

To further assess the effectiveness of metaphor feature sets, we compared metaphor-based feature set and sentiment-based feature set with three common text features that are extracted by LIWC, NRC Emotion Lexicon, and VADER Sentiment Lexicon and used in the logistic regression baseline method. The line charts shown in Figure 4 present the accuracy and F1-score performance of each feature separately for prediction of the six mental health problems using the neural network classifier. The results show that metaphor feature sets are more effective at predicting inferiority and sensitivity than other textual features and equally effective at predicting other mental health problems.

## 6. Conclusions

To the best of our knowledge, we are the first to demonstrate the prediction of six mental problems—anxiety, depression, inferiority, sensitivity, social phobias, and obsession—using automatically detected metaphors in texts. We used metaphor-based feature sets and sentiment-based feature sets to predict these mental health problems using a compositional dataset produced by second-language students and the eRisk2017 dataset collected from Social Media. Our results show that the proposed method can predict the mental health status of authors of written texts, and our algorithm performs well compared to other state-of-the-art methods. We also analyzed differences in metaphor use among students with various mental health problems and evaluated the effectiveness of metaphor sets compared with other textual features in predicting mental health status from a compositional dataset of second-language students.

Our work demonstrates the value of metaphorical textual features for the prediction of mental health problems. The experiment results remind us of the importance of metaphor, as a deep, complex, and cognitive feature for mental health identification, which often focuses on shallow linguistic features. Importantly, we show that metaphor is predictive even for nonnative speakers of the language. We also contribute to a novel, scarce, and valuable dataset, consisting of second-language speakers' essays and data on authors' mental health problems obtained from a psychological survey, which we will release publicly. We hope this paper will stimulate new ideas for the identification and prediction of mental health status through analysis of text and lead to improvement of automated methods for this purpose.

## Figures and Tables

**Figure 1:** The figure of our work flow.

**Figure 2:** Metaphor examples identified by automatic metaphor identification method.

**Figure 3:** The characteristic of metaphor usage of each mental illness. (a) The probability of sentence with metaphor. (b) The number of positive metaphor. (c) The number of negative metaphor. (d) The average sentiment score of metaphor.

**Figure 4:** Accuracy and F1-score of every feature separately on six mental illness prediction tasks.

**Algorithm 1:** Framework of feature set generation for MSM.

**Algorithm 2:** Metaphor identification algorithm.

**Table 1:** Mental health data of students.

Problem	No. of students	Problem	No. of students
Anxiety	36	Sensitivity	49
Depression	36	Social phobia	44
Inferiority	29	Obsession	38
One problem	28	Two problems	21
Three problems	21	Four problems	10
Five problems	7	Six problems	7

*N* problems mean the students with *n* mental problems at the same time.

**Table 2:** The examples of frequent metaphors in each state of mind.

Mental problem	Frequent metaphor	Example sentence
Anxiousness	Hit, present, join	The poor of property can't hit me, but a boring life can
Depression	Chase, clean, tough	Maybe there will be many difficulties in the way I chase my dream
Inferiority	Support, independent	All these support his spirit of “learning insatiably”
Sensitivity	Defeat, move, create	I know in this process some trouble will defeat me
Social phobia	Raise, affect, stop	It is really a burden for a poor family to raise a child
Obsession	Enter, guide, control	When you enter the society, you probably have problem in finding a job
Healthy control	Develop, pass, lead	I want to develop a wonderful game

**Table 3:** The statistical information of emotion in various mental states.

Mental state	Anxiousness	Depression	Inferiority	Sensitivity	Social Phobia	Obsession	Healthy control	Total
Avg. emotion	0.118	0.129	0.110	0.159	0.083	0.038	0.129	0.129
Meta emotion	0.047	0.100	0.066	0.118	0.033	0.036	0.079	0.079

**Table 4:** Prediction performance on the eRisk 2017 dataset.

Method		Accuracy	F1-score
Trotzek et al.	CNN	0.88	0.59
	LR	0.88	0.69

MSM	Sentiment	0.81	0.61
	Metaphor	0.87	0.56
	ALL	0.89	0.70

All: sentiment + metaphor.

**Table 5:** Accuracy of baseline and MSM on six mental illnesses' prediction.

Method	Trotzek et al.		MSM		
	CNN	LR	All	Sent	Meta
Anxiousness	0.75	0.71	**0.82**	0.61	0.71
Depression	0.73	0.69	**0.75**	0.63	0.70
Inferiority	0.78	0.72	0.80	0.80	**0.85**
Sensitivity	0.58	0.62	**0.80**	0.53	0.78
Social phobia	0.64	0.65	**0.71**	0.60	0.70
Obsession	0.68	0.74	**0.78**	0.72	0.75
Average	0.69	0.69	**0.78**	0.65	0.75

Sent: sentiment-based feature set; meta: metaphor-based feature set; all: sent + meta.

**Table 6:** F1-score of baseline and MSM on six mental illnesses' prediction.

Method	Trotzek et al.		MSM		
	CNN	LR	All	Sent	Meta
Anxiousness	0.57	**0.65**	0.64	0.51	0.54
Depression	0.50	0.64	**0.67**	0.51	0.58
Inferiority	0.46	0.63	0.62	0.51	**0.71**
Sensitivity	0.46	0.59	**0.73**	0.44	0.70
Social phobia	0.47	0.61	0.58	0.50	**0.62**
Obsession	0.42	**0.69**	0.66	0.50	0.59
Average	0.48	0.64	**0.65**	0.50	0.62

Sent: sentiment-based feature set; meta: metaphor-based feature set; all: sent + meta.

## Data Availability

The data used to support the findings of the study are available from the corresponding author upon request.
